The article "Identification of Key Biomarkers and Immune Infiltration in Liver Tissue after Bariatric Surgery" was retracted in 2023. Reasons: unreliable results or conclusions; concerns about the data; concerns about the peer review; concerns about the citations.

# Identification of Key Biomarkers and Immune Infiltration in Liver Tissue after Bariatric Surgery

**DOI:** 10.1155/2022/4369329

**Published:** 2022-06-25

**Authors:** Xiaoyan Zhang, Jingxin Li, Tiancai Liu, Min Zhao, Baozhu Liang, Hong Chen, Zhen Zhang

**Affiliations:** ^1^Department of Endocrinology and Metabolism, Zhujiang Hospital, Southern Medical University, Guangzhou, China; ^2^Department of Pediatrics, Guangdong Provincial People's Hospital, Guangdong Academy of Medical Sciences, Guangzhou, China; ^3^School of Laboratory Medicine and Biotechnology, Institute of Antibody Engineering, Southern Medical University, Guangzhou, China

## Abstract

**Background:**

Few drugs are clearly available for nonalcoholic fatty liver disease (NAFLD) and nonalcoholic steatohepatitis (NASH); nevertheless, mounting studies have provided sufficient evidence that bariatric surgery is efficient for multiple metabolic diseases, including NAFLD and NASH, while the molecular mechanisms are still poorly understood.

**Methods:**

The mRNA expression profiling of GSE48452 and GSE83452 were retrieved and obtained from the Gene Expression Omnibus (GEO) database. The limma package was employed for identifying differentially expressed genes (DEGs), followed by clusterProfiler for performing Gene Ontology (GO) and Kyoto Encyclopedia of Genes and Genomes (KEGG) analyses, and GSEA software for performing GSEA analyses. The PPI network analyses were constructed using Metascape online analyses. WGCNA was also utilized to identify and verify the hub genes. CIBERSORT tools contributed to the analysis of immune cell infiltration of liver diseases.

**Results:**

We identify coexpressed differential genes including 10 upregulated and 55 downregulated genes in liver tissue after bariatric surgery. GO and KEGG enrichment analyses indicated that DEGs were remarkably involved in the immune response. GSEA demonstrated that DEGs were markedly enriched in the immune response before surgery, while most were enriched in metabolism after surgery. Seven genes were screened through the MCC algorithm and KME values, including SRGN, CD53, EVI2B, MPEG1, NCKAP1L, LCP1, and TYROBP. The mRNA levels of these genes were verified in the Attie Lab Diabetes Database, and only LCP1 was found to have significant differences and correlation with certain immune cells.

**Conclusion:**

Our knowledge of the mechanisms by which bariatric surgery benefits the liver and the discovery of LCP1 is expected to serve as potential biomarkers or therapeutic targets for NAFLD and NASH.

## 1. Introduction

There is considerable evidence that nonalcoholic fatty liver disease (NAFLD), which is widespread around the world, affects about one in four adults [1]. NAFLD encompasses a series of histological findings, including simple steatosis, steatohepatitis, and cirrhosis. The former contains at least 5% hepatic steatosis without hepatocyte ballooning, meanwhile excluding liver disease induced by excessive alcohol intake, while NASH involves at least 5% hepatocyte steatosis and inflammation with hepatocellular injury (e.g., ballooning), with or without fibrosis [2]. NAFLD not only causes chronic disorders of the liver, for instance, cirrhosis and hepatocellular carcinoma, but also is highly correlated with numerous systemic metabolic diseases, including type 2 diabetes, overweight/obesity, and hypertension [3–6]. The high incidence of such liver disease is associated with a rapid increase in sedentary behavior, decrease in physical activity, and excessive calorie consumption resulting from nutritional and diet imbalances [7].

The article "Identification of Key Biomarkers and Immune Infiltration in Liver Tissue after Bariatric Surgery" was retracted in 2023. Reasons: unreliable results or conclusions; concerns about the data; concerns about the peer review; concerns about the citations.

In view of the increased understanding of the pathogenesis and rising incidence of NAFLD, experts have recently proposed the clinical diagnosis, namely, metabolic dysfunction-associated fatty liver disease (MAFLD). The reference standard of diagnosis is evidence of hepatic fat accumulation (hepatic steatosis) based on histology, imaging data, or blood biomarkers, with one of the following three conditions: overweight/obesity, type 2 diabetes (T2DM), or other metabolic disturbances [8]. Overweight or obesity has shown a strong and consistent pathological association with MAFLD and has been a crucial determinant of adverse clinical outcomes, for which it becomes one of the main criteria for defining MAFLD [8]. A large cohort study suggested that obesity was independently associated with NAFLD regardless of metabolic profiles [9]. A recent study confirmed that obese patients also had a higher fatty liver activity score (NAS) and increased incidence of hepatocellular ballooning (a marker of liver inflammation), together with accelerated fibrosis progression rates compared to nonobese patients [10].

Given the lack of approved drug treatments for MAFLD, targeted treatment of obesity through lifestyle changes remains an essential measure and a reasonable treatment option for the management of MAFLD [11], which, however, is indeed challenging to achieve and maintain. Studies have proposed that only weight loss of ≥3% can improve steatosis, ≥5% can improve inflammation, and ≥10% can improve fibrosis, which is difficult to achieve with lifestyle interventions [12, 13].

Additional medications are recommended when lifestyle interventions fail. Several drugs have been performed in clinical tests, but there are no widely recognized drug treatments for NAFLD and NASH yet. Pioglitazone was proven to improve histology of liver in steatosis, inflammation, and hepatocyte ballooning, enhancing NASH and fibrosis remission [14]. Nevertheless, NASH recurred after withdrawal as serum alanine aminotransferase levels increased. There is also a concern about a weight-gain problem with taking pioglitazone [14, 15]. PIVENS results suggested that vitamin E could improve histology in NASH, but chronic use might be relevant to increasing the risk of hemorrhagic strokes as well as prostate cancer [16, 17]. Liraglutide, a promising drug in phase 2 clinical trials currently, has relatively few side effects in addition to its beneficial effects in treating NAFLD [18, 19]. Obeticholic acid (OCA) has progressed to phase 3 development for NASH, which has potential effects in terms of attenuating liver steatosis and inflammation as well as fibrosis, meanwhile increasing insulin sensitivity. In a phase 2 trial, patients treated with OCA had a ≥2-point reduction in NAS with no exacerbation of fibrosis, although there was some evidence of exacerbation of dyslipidemia, which could be ameliorated with a combination of statins [20]. In summary, no single drug or combination has been widely recognized to be effective for patients with NASH, despite the initial evaluation of numerous agents.

The article "Identification of Key Biomarkers and Immune Infiltration in Liver Tissue after Bariatric Surgery" was retracted in 2023. Reasons: unreliable results or conclusions; concerns about the data; concerns about the peer review; concerns about the citations.

As recommended by AASLD [21], EASL/EASD/EASO [22], and APWP [23] guidelines, bariatric surgery might be accepted for particular morbidly obese patients with NAFLD who fail to respond to lifestyle-adjusting and pharmaceutical interventions. This is because bariatric surgery is proven to be the most efficient means of working to sustain long-term weight reduction, which not only is beneficial for NAFLD but also reduces chronic mortality associated with heart disease, diabetes, and cancer [24, 25]. The surgical effects extend far beyond the demonstrably major goal of weight reduction to metabolic improvement further, thus being figuratively called “metabolic surgery.” Accompanied by continuing improvements in the last decades, bariatric surgery has stepped into the era of laparoscopic surgery. With this background, Roux-en-Y gastric bypass (RYGB) has been universally regarded as the preferred choice, and other types include LAGB, SG, VGB, or mixed [26]. As reported by Mummadi et al., results from liver biopsies showed improvement or regression rates of 91.6%, 81.3%, and 65.5%, respectively, in steatosis, steatohepatitis, and fibrosis after bariatric surgery [27]. Another meta-analysis targeting 21 studies and 2374 patients also proposed that bariatric surgery ameliorated or alleviated steatosis in 88% of patients, steatohepatitis in 59% of patients, and fibrosis in 30% of patients. Compared with other surgical types, RYGB seems to play a larger role in the regression or improvement of histological features of NAFLD, although there is a lack of consistency in biochemical manifestations [28]. Indeed, a majority of studies have shown that bariatric surgery is relevant to remarkable reductions in biochemical criteria such as ALT, AST, ALP, and GGT [29]. It is interesting to note that patients treated with RYGB showed a remarkable decrease in liver lipid capacity and improvement in liver insulin sensitivity prior to appreciable weight reduction [30, 31].

The article "Identification of Key Biomarkers and Immune Infiltration in Liver Tissue after Bariatric Surgery" was retracted in 2023. Reasons: unreliable results or conclusions; concerns about the data; concerns about the peer review; concerns about the citations.

To the best of our knowledge, these liver benefits are at least directly associated with the intestinal peptide GLP-1 and peptide YY (PYY) [32, 33]. Dixon et al. found that NASH occurred in only 10% of patients at 29.5 months of follow-up biopsies after LAGB, and all patients had improvement in steatosis, inflammation, and fibrosis and biochemical markers for liver function [34, 35]. Furthermore, researchers concluded that a reduction in gamma-glutamyltransferase concentration might be related to histological improvement [34, 35]. Pournaras et al. observed elevated concentrations of bile acids, FGF19, incretin, and satiety intestinal hormone after gastric bypass surgery, while elevated FGF19 and reduced Ghrelin concentrations may contribute to the improvement of inflammation and biochemical indicators after gastric bypass surgery to a certain extent [36]. In addition, bile acids may participate in the alterations in energy homeostasis caused by bariatric surgery through the following two mechanisms: (1) increased secretion directly affects energy balance; (2) nutrient and bile diversion leads to increased transport to the distal intestine, stimulating the hormone production and release of L cells to weaken the effect of bariatric surgery [37].

NAFLD is a typical heterogeneous disease involving multiple pathogenic pathways [38]. One dominant theory proposes that accumulated triglycerides induce cellular damage caused by oxidative stress, protein misfolding, mitochondrial damage, and endoplasmic reticulum stress responses [39], leading to a persistent state of chronic inflammation that directs body tissue toward immunity and inflammation overactivation [40]. It has been suggested that both innate and adaptive immune activation can further trigger and magnify liver inflammation during the occurrence and progression of NAFLD/NASH [41, 42], referring to the activation of resident Kupffer cells and recruitment of white blood cells such as neutrophils, dendritic cells, and CD8+ T cells [43–46]. Haas et al. also reported that NASH activity was associated with changes in blood immune cell populations, including conventional dendritic cell (cDC) subpopulations and CD8 T cells. They found increased expression of NASH transcriptional characteristic genes in the liver and altered CDC and CD8 T cell numbers in obesity-driven NASH mouse models [47]. These results suggest that different immune cell populations play an important role in the pathogenesis of NASH and therefore are expected to be potential therapeutic targets for NASH. More notably, differentiation of CD4+ T cells into helper T cells type17 (TH17) in response to inflammatory stimuli was found to be associated with progression of NAFLD to NASH, and these changes appeared to return to normal 1 year after bariatric surgery [48, 49]. The reduction of nutritional metabolites regulated by bariatric surgery is likely to promote the development of anti-inflammatory status and metabolic function by inhibiting pathological immune responses [50]. However, the more detailed relationship between bariatric surgery and NASH immune status remains to be explored. In summary, further research is required to confirm its curative effect and potential mechanisms before bariatric surgery can be recommended as an approach to treat NASH.

The article "Identification of Key Biomarkers and Immune Infiltration in Liver Tissue after Bariatric Surgery" was retracted in 2023. Reasons: unreliable results or conclusions; concerns about the data; concerns about the peer review; concerns about the citations.

With rapid advances in high-throughput sequencing technology, bioinformatics analysis techniques have become a prospective method to investigate the underlying mechanisms of surgical benefit. We determined DEGs in liver tissue of the postoperative group by analyzing mRNA expression profiles searched and obtained from the GEO database. Afterwards, Gene Ontology (GO), Kyoto Encyclopedia of Genes and Genomes (KEGG), and GSEA were used to investigate the underlying mechanisms for surgical benefit. Next, we built a PPI network, then utilized CytoHubba in Cytoscape and modular information in WGCNA analysis to identify hub genes, which were verified in the Attie Lab Diabetes Database. Finally, the “ggplot2” package was applied to visualize the differences between preoperative and postoperative groups in immune cell infiltration, which was also utilized to analyze the correlations between hub genes and infiltrating immune cells. Our knowledge of the mechanisms by which bariatric surgery benefits the liver and the discovery of LCP1 is expected to serve as potential biomarkers or therapeutic targets for NAFLD and NASH.

## 2. Materials and Methods

### 2.1. Microarray Data Acquisition and Processing

Microarray profiles GSE83452 and GSE48452 were searched and extracted in the GEO (http://www.ncbi.nlm.nih.gov/geo) database with search strategy (bariatric surgery [All Fields] and liver tissue [All Fields]) and (“Homo sapiens” [Organism] and “Expression profiling by array” [filter]).

The article "Identification of Key Biomarkers and Immune Infiltration in Liver Tissue after Bariatric Surgery" was retracted in 2023. Reasons: unreliable results or conclusions; concerns about the data; concerns about the peer review; concerns about the citations.

Inclusion criteria were as follows: (i) Liver tissue from obese patients diagnosed downgrading by liver biopsy at 1-year follow-up after bariatric surgery. (ii) Liver tissue from obese patients diagnosed with NAFLD or NASH by liver biopsy at baseline served as controls. We downloaded the preprocessing matrix data of GSE83452 and GSE48452 and converted the data at the probe level to the data at the gene level. Lastly, eight preoperative samples, eight corresponding postoperative samples, and 18,084 common genes were obtained from GSE48452 (platforms: GPL11532, [HuGene-1_1-st] Affymetrix Human Gene 1.1 ST Array [transcript (gene) version]). Meanwhile, thirteen preoperative samples, thirteen corresponding postoperative samples, and 15,399 common genes were obtained from GSE83452 (platforms: GPL16686, [HuGene-2_0-st] Affymetrix Human Gene 2.0 ST Array [transcript (gene) version]).

### 2.2. Identification of Differentially Expressed Genes

DEGs in liver tissue of postoperative samples were screened out by performing the limma V3.42.0 package with criteria of |log *FC*| > 0.5 and adj *P* < 0.05. The Sangerbox3.0 online tool was applied to draw the volcano and Venn diagrams, and the overlapping DEGs of two datasets were retained for further analysis.

### 2.3. Functional and Pathway Enrichment Analysis

To annotate the overlapping DEGs in terms of function and pathway, we used clusterProfiler (Version 3.14.3) for GO terms and KEGG analysis by taking the GO annotations (version 3.1.0) and the latest KEGG pathway annotations as the background. The above results were displayed in a bar graph and circle graph, respectively (http://soft.sangerbox.com/).

### 2.4. Gene Set Enrichment Analysis

We downloaded GSEA software from the GSEA website (http://software.broadinstitute.org/gsea) and the subset (C2.cp.kegg.v7.4.Symbols.gmt) from the Molecular Signatures Database. The samples were divided into two groups according to before and after bariatric surgery. Then, GSEA analysis was utilized to investigate the underlying pathways and molecular mechanisms. The random combinations were set to 1000 times. Results that met the conditions of *P* < 0.05 and FDR < 0.25 were recognized as significant.

### 2.5. Construction of PPI Network

DEGs were entered into the Metascape database (http://metascape.org) for protein-protein interaction enrichment analysis, in which all interactions in STRING (combined score > 0.187) were used, and the Molecular Complex Detection (MCODE) algorithm10 was performed to recognize network components at tight junctions. Next, Cytoscape software was utilized to visualize the PPI network for DEGs.

### 2.6. Construction of Weighted Gene Coexpression Network Analysis (WGCNA)

The WGCNA package in R software was carried out to construct a common expression network for differentially expressed genes. On the basis of the principle of a scale-free network, a weighted adjacency matrix was built and the soft threshold parameter was determined. Next, we transformed the adjacency matrix into the topological overlap matrix (TOM), which was utilized to reduce noise and false correlation. Then, hierarchical cluster analysis was applied to obtain different gene modules. Then, we evaluated the correlation between modules and phenotypes, and the one of most interest that is closely associated with clinical traits was determined.

The article "Identification of Key Biomarkers and Immune Infiltration in Liver Tissue after Bariatric Surgery" was retracted in 2023. Reasons: unreliable results or conclusions; concerns about the data; concerns about the peer review; concerns about the citations.

### 2.7. Identification and Validation of Hub Genes

Firstly, CytoHubba, a plug-in of Cytoscape, was employed to screen the hub genes existing in the PPI network constructed based on DEGs with the MCC algorithm, which had consistently exhibited a satisfying comparative performance. Secondly, for WGCNA analysis, hub genes appear to be those with high KME (eigengene connectivity) values, that is, with the most links in the network. Thus, the hub genes of the module of interest in the GSE48452 database were screened on the condition that KME values were greater than 0.9 (*P* < 0.05). The hub genes were also identified by KME > 0.9 in the GSE83452 database. At last, the genes screened by these methods were visualized as a Venn diagram to determine the overlapping ones, of which we verified the mRNA levels in Attie Lab Diabetes Database (*P* < 0.05 was set as significant).

### 2.8. Evaluation of Immune Cell Infiltration

We load the official source of CIBERSORT (https://cibersort.stanford.edu/) in the RStudio code and the specified benchmark database file (LM22.txt, which is the marker gene of 22 immune cells). Imported gene expression profile data were utilized to analyze and summarize the proportion of immune cells, where permutations for significance analysis were set to 1000 times, and then, the proportion of 22 types of immune cell infiltration corresponding to each sample was obtained. The results were then visualized using the “ggplot2” package to draw violin plots and heat maps. The “corrplot” package (https://CRAN.R-project.org/package=corrplot) was applied to draw a heat map of correlations between infiltrating immune cells.

### 2.9. Correlation Analysis between Hub Gene and Infiltrating Immune Cells

Spearman correlation analysis was performed on hub genes and immune infiltrating cells with the “psych” package (https://CRAN.R-project.org/package=psych), and the “ggplot2” package was used to draw lollipop plots for visualization of the results.

## 3. Result

### 3.1. DEG Screening and Identification after Bariatric Surgery

The gene expression matrix of the two groups was presented in a two-dimensional PCA cluster diagram (Figures 1(a) and 1(d)). The results showed that the two groups of samples had obvious clustering, indicating that the source of samples was reliable. Then, 589 and 251 DEGs were screened from GSE48452 and GSE83452 according to defined criteria (|*logFC*| > 0.5 and adj *P* < 0.05), respectively. DEGs were demonstrated with a volcano map (Figures 1(b) and 1(e)) and heat map (Figures 1(c) and 1(f)), which were clustered via Euclidean distance. GSE48452 included 204 upregulated genes and 385 downregulated genes, while GSE83452 contained 65 upregulated genes and 186 downregulated genes. The coexpressed DEGs were presented with a Venn graph online tool, containing 10 upregulated (Figure 1(g)) and 55 downregulated (Figure 1(h)) genes in liver tissue.

The article "Identification of Key Biomarkers and Immune Infiltration in Liver Tissue after Bariatric Surgery" was retracted in 2023. Reasons: unreliable results or conclusions; concerns about the data; concerns about the peer review; concerns about the citations.

### 3.2. Gene Ontology and KEGG Pathway Enrichment Analyses of DEGs

To annotate the overlapping DEGs in terms of function and pathway, we used clusterProfiler (version 3.14.3) to perform GO annotation and KEGG analysis. The result of GO terms revealed that for BP analysis, DEGs after bariatric surgery were mainly enriched in the immune system process, response to external stimulus, and response to stress (Figure 2(a)). Regarding CC, the overlapping DEGs were significantly enriched in transcription factor AP-1 complex, plasma membrane part, and external side of plasma membrane (Figure 2(a)). MF analysis showed that cargo receptor activity, proteoglycan binding, and RNA polymerase II activating transcription factor binding are the most prominent GO terms (Figure 2(a)). KEGG enrichment analysis demonstrated that fluid shear stress and atherosclerosis were a noteworthy pathway (Figure 2(b)).

### 3.3. GSEA Analysis

To evaluate deeply the pathways and molecular mechanisms involved, samples were divided into two groups according to before and after bariatric surgery; then, GSEA analysis was performed on GSE48452 and GSE83452. The final results highlighted that the most prominent gene sets showed positive correlations with the preoperative group, including graft versus host disease, allograft rejection, type I diabetes mellitus, and intestinal immune network for IGA production in both GSE48452 and GSE83452 (Figures 2(c) and 2(d)), containing hematopoietic cell linage, antigen procession, and presentation in GSE48452 (Figure 2(c)) and autoimmune thyroid disease and leishmania infection in GSE83452 (Figure 2(d)). Additionally, the most remarkably enriched gene sets that display positive correlations with the postoperative group in GSE83452 were Huntington's disease, the Notch signaling pathway, and glycine serine and threonine metabolism (Figure 2(e)).

The article "Identification of Key Biomarkers and Immune Infiltration in Liver Tissue after Bariatric Surgery" was retracted in 2023. Reasons: unreliable results or conclusions; concerns about the data; concerns about the peer review; concerns about the citations.

### 3.4. PPI Network Analysis

As shown in Figure 3(a), we input overlapping DEGs into the Metascape database for PPI network construction and obtain 4 major different modules, in which genes are at tight functions. To make it easier to describe next, we used red, blue, green, and purple colors to represent them. Moreover, we performed enrichment analysis on each MCODE component, retaining and displaying three terms with the lowest *P* value score to describe the functions of the component, defined in Figure 3(b), containing immune response-regulating signaling pathway in red MCODE, leukocyte cell-cell adhesion in blue MCODE, low-density lipoprotein particle clearance in green MCODE, and transcription factor AP-1 complex in purple MCODE, etc.

### 3.5. Construction of WGCNA and Identification of Interested Module

The WGCNA package in R software was carried out to build a coexpression network for DEGs. We calculated the correlation between gene modules and phenotypes with the Pearson method, and the obtained results were visualized with heat maps (Figure 4(a)). It turned out that only the red module met the criteria for a strong correlation not only with bariatric surgery but also with fat, inflammation, and NAS. That is to say, the red module is highly related to bariatric surgery as well as the occurrence of fat, inflammation, and NAS in NAFLD patients. Besides, the relationship between phenotype features and the red module as well as gene expression was presented with a vector graph (Figure 4(b)). The higher the correlation in Figure 4(b) indicates the higher consistency between the genes in the module and the eigenvector of the module, further confirming that the genes in the red module are highly related to the above phenotypes. Therefore, we will focus on studying and analyzing the detailed information of genes in the red module.

### 3.6. Identification and Validation of Hub Genes

First, 65 differentially expressed genes that overlapped in the two datasets were classified into the PPI network through protein functional enrichment of the STRING website. *MPEG1*, *TYROBP*, *RGS1*, *SRGN*, *PLEK*, *CD53*, *THEMIS2*, *LAPTM5*, *NCKAP1L*, *EVI2B*, *CTSS*, *CD84*, *LCP1*, *JUN*, *ANXA5*, *FOS*, *PECAM1*, *IGF1*, *CD163*, *FPR3*, *VSIG4*, *SGK1*, *DDIT4*, *GDF15*, *MSN*, *AOAH*, *JUND*, *JUNB*, *TXNIP*, and *RHOB* were the top 30 genes according to the MCC algorithm in CytoHubba of Cytoscape.

The second step was to screen genes based on the condition that KME values were greater than 0.9 (*P* < 0.05) of the module of interest, namely, the red module in the GSE48452 database, producing 53 hub genes thus. In addition, the darkorange2 module was determined as the module of interest in GSE83452, as it had the strongest negative correlation with bariatric surgery, in which 14 hub genes were also identified according to defined criteria (KME > 0.9).

The article "Identification of Key Biomarkers and Immune Infiltration in Liver Tissue after Bariatric Surgery" was retracted in 2023. Reasons: unreliable results or conclusions; concerns about the data; concerns about the peer review; concerns about the citations.

Finally, the hub genes determined by the aforementioned three means are visualized as a Venn graph, as shown in Figure 5(a), including *SRGN*, *CD53*, *EVI2B*, *MPEG1*, *NCKAP1L*, *LCP1*, and *TYROBP*. We utilized Attie Lab Diabetes Database to validate the mRNA levels of the above-mentioned genes in obese mice, except SRGN which was lacking in the database (Figure 5(b)). The results demonstrated that LCP1 expression was remarkably upregulated in obese mice at 4 and 10 weeks compared with the lean group.

### 3.7. Immune Cell Infiltration Results

Using the CIBERSORT algorithm, we first explored the differences in immune infiltration of liver tissues between the postoperative and the preoperative in 22 immune cell subpopulations. The violin plots of the immune cell infiltration difference in GSE83452 indicated that (Figure 6(a)), compared with the preoperative group, the postoperative group generally contained a lower proportion of M1 macrophages (*P* = 4.2*e* − 03). An accumulative bar diagram was performed to further visualize the relative proportions of immune cells in each sample of GSE83452 (Figure 6(c)) datasets. Correlation heat map of immune cells revealed changes in the correlation between immune cells in the samples before and after surgery. The multiple correlations between immune cells present in the preoperative samples (Figure 6(b)) disappeared or changed in the postoperative samples. For example, activated NK cells were significantly positively correlated with resting Mast cells in preoperative samples (*P* < 0.001), while the correlation was absent in postoperative groups.

### 3.8. Correlation Analysis between LCP1 and Infiltrating Immune Cells

As shown in Figure 6(d), results from GSE83452 revealed that LCP1 were positively correlated with M1 macrophages and memory B cells (*P* < 0.05), while negatively correlated with regulatory Tregs and CD8 T cells (*P* < 0.05), suggesting that LCP1 was remarkably associated with both innate immunity (macrophages, NK cells, etc.) and adaptive immune system (B cells and various types of T cells), both of which participated in the pathogenesis of NAFLD/NASH.

## 4. Discussion

As mentioned before, NAFLD has been found to be one of the most prevalent chronic liver diseases (with a global incidence of approximately 25% of the adult population) [1], which was also considered to have a strongly bidirectional connection to components of the metabolic syndrome [51]. NAFLD is a heterogeneous disease with varying rates of progression and clinical outcomes [4], involving multiple pathogenicity pathways regulated by a variety of metabolic, genetic, and microbiome-related factors, which are not entirely known today [52]. Overnutrition is believed to be a major driver of NAFLD, leading to the expansion of fat depot and the accumulation of heterotopic fat. In this case, the proinflammatory state produced by the infiltration of macrophages between visceral adipose tissues promotes insulin resistance. Then, improper lipolysis in response to insulin resistance results in an imbalance of lipid metabolism and accumulation of lipotoxic lipids that create cellular stress, inflammasome activation, and apoptotic cell death, subsequently stimulating inflammation, tissue regeneration, and fibrosis [53, 54]. There is some evidence suggesting that surgical weight-loss remarkably improves metabolic dysfunction, contributing to alleviating the occurrence and development of NAFLD/NASH [55]. However, the underlying mechanism by which bariatric surgery promotes remission of NAFLD/NASH remains unclear to some extent.

The article "Identification of Key Biomarkers and Immune Infiltration in Liver Tissue after Bariatric Surgery" was retracted in 2023. Reasons: unreliable results or conclusions; concerns about the data; concerns about the peer review; concerns about the citations.

Against this background, integrated bioinformatics methods based on two GEO datasets, namely, GSE48452 and GSE83452, helped to analyze the changes in gene expression levels after bariatric surgery to reveal potential pathways that attenuated liver tissue steatosis and inflammation and identified the total overlapping 65 DEGs, including 55 downregulated DEGs and 10 upregulated DEGs.

Further enrichment analyses were applied to elucidate the primary action of overlapping DEGs. BP analysis in GO terms suggested that DEGs were mainly enriched in the immune system process, response to external stimulus, and response to stress. Previous studies have indicated that NASH hepatocyte injury was characterized by endoplasmic reticulum (ER) stress [56], dysfunctional unfolded protein responses [57], inflammasome activation [58], apoptotic pathway activation, inflammation, and enhanced trauma responses [59].

For NAFLD/NASH, innate immune activation is a critical factor in triggering and amplifying liver inflammation [41], and the occurrence of the former involves the activation of resident Kupffer cells [43, 60] and recruitment of white blood cells such as neutrophils, dendritic cells, natural killer cells (NK), and natural killer T cells (NKT) [44, 45, 61, 62], which facilitated the inflammatory responses by releasing cytokines, chemokines, eicosane compounds, nitric oxide, and reactive oxygen species [53, 63]. Adaptive immunity is another significant factor in contributing to liver inflammation [42]. Liver infiltration of B, CD4+, and CD8+ T cells was evident in varying NASH models, parallel to worsening parenchymal damage and lobular inflammation. In response to inflammatory stimuli, CD4+ T cells can also differentiate into helper T cells type 17 (TH17), the accumulation of which was found to be associated with progression from NAFLD to NASH, and interestingly, these changes appear to go back to normality at 1 year after bariatric surgery, along with improvements in liver inflammation [46, 48, 63–65]. Therefore, it is reasonable to infer that bariatric surgery is likely to alleviate stress and inflammation by acting on the regulation of immune function, thereby reducing liver cell damage. More details will be discussed later.

The article "Identification of Key Biomarkers and Immune Infiltration in Liver Tissue after Bariatric Surgery" was retracted in 2023. Reasons: unreliable results or conclusions; concerns about the data; concerns about the peer review; concerns about the citations.

The previous result is consistent with the CC analysis, showing that the transcription factor AP-1 complex is one of the most significant GO terms. The AP-1 complex, composed of members of the Fos and Jun families, has an impressive impact on cell proliferation and neuronal activation, meanwhile involving cell stress-induced apoptosis, DNA damage agents, or the absence of survival signals [66–68], which undoubtedly occurs in the disease development of NASH. Moreover, MF analysis showed that DEGs are prominently enriched in cargo receptor activity, proteoglycan binding, and RNA polymerase II activating factor binding. KEGG analysis demonstrated that fluid shear stress and atherosclerosis was a significant pathway.

GSEA was performed to clarify a novel insight for this research. It has indicated that surgically caused weight reduction leads to a shift in NAFLD/NASH from a proinflammatory to an anti-inflammatory state, thus resulting in metabolism improvement. GSEA demonstrated that most genes in preoperative subjects were primarily enriched in graft versus host disease, allograft rejection, type I diabetes mellitus, intestinal immune network for IGA production, antigen procession and presentation, autoimmune thyroid disease, and so on.

Rejection is caused by recipient T cells recognizing alloantigens of nonself-donors, the overall effect of which is to induce a proinflammatory microenvironment in the liver of allograft, contributing to tissue damage [69]. The specific mechanism underlying the effects have been confirmed to include activation of Kupffer cells; the release of proinflammatory cytokines like TNF, IFN, IL-1, and IL-12; recruitment of neutrophils to the graft [70]; alloantigen presentation of dendritic cells [71]; and activation, maturation, and migration of CD4+ and CD8+ cells to the liver [72–74]. In addition, donor-specific antibodies (DSA) may drive antibody-mediated rejection through the differentiation of activated B cells into plasma cells and the initiation of DSA production. Other cells migrate to the lymph node that forms the germinal center and undergoes a process of somatic maturation that refines and amplifies antibody responses [75]. Hence, it could be concluded that the role of innate and adaptive immunity shares a number of similarities in NAFLD/NASH (as previously described) and in allograft rejection. Type 1 diabetes mellitus and autoimmune thyroiditis are the most common immunologic endocrine disorders, which result from autoimmune-mediated tissue destruction, similarly involving a mechanism of activation and maturation of T cells [76]. There have been numerous studies on immunosuppressive therapy for these diseases. Do these findings have any reference for the treatment of NAFLD/NASH? It is worth contemplating and exploring. It should be noted that the degree of influence of drugs on liver fibrosis is an additional aspect to take into account in this regard.

The article "Identification of Key Biomarkers and Immune Infiltration in Liver Tissue after Bariatric Surgery" was retracted in 2023. Reasons: unreliable results or conclusions; concerns about the data; concerns about the peer review; concerns about the citations.

In addition, GSEA indicated that most genes in postoperative subjects were primarily enriched in glycine, serine, and threonine metabolism. Previous studies have shown that metabolites that primarily maintain metabolic functions, such as fatty acids, glucose, and amino acids, could regulate the function and metabolism of immune-related cells [77]. It is therefore very likely that the reduction of nutritional metabolites regulated by bariatric surgery leads to advances in anti-inflammatory status and metabolic function by inhibiting pathological immune responses [50].

We applied the MCODE algorithm to recognize the network components at tight junctions in the PPI network, in which we then carried out enrichment analysis. The results also highly suggested that the function of the component was closely related to the immune response, which was consistent with our previous GO functional enrichment and GSEA analysis results.

Currently, remission of NASH (no progression of fibrosis) and/or improvement of fibrosis (no deterioration of NASH) have been the regulatory-approved endpoint in clinical trials, which is thus the criteria for establishing a novel therapeutic approach. On the one hand, performing the development and validation of novel noninvasive methods to investigate the fibrosis progression or resolution of NASH will promise to help advance the therapy of NAFLD/NASH [78]. On the other hand, with the continuous disclosure of new information on the pathogenesis of NAFLD/NASH, numerous pathogenic factors (insulin resistance, lipid toxicity, oxidative stress, changes in immune/cytokine/mitochondrial function, and apoptosis) are found associated with the occurrence and progression of NASH [79]. The development of one or more combination therapies that can improve both NASH and fibrosis is the major direction of future efforts to address NAFLD/NASH diseases. Preventing or addressing simple steatosis may be a promising measure to interfere with the follow-up progression of NASH [80]. Steatosis can be graded by the frequently utilized NAFLD Activity Score (NAS), which is used additionally to assess inflammation and hepatocyte damage. Results indicated that activity levels tended to decrease with fibrosis regression, despite the persistence of steatohepatitis, while increased activity levels were correlated with fibrosis progression [81, 82]. With the WGCNA analysis, we identified that the red modules, possessing a significantly negative correlation with bariatric surgery, were highly correlated with fat, inflammation, and NAS. Although there is no immediate significant evidence of a direct relationship between red module and fibrosis, pharmacological intervention and observational research have displayed the same direction between activity levels, liver inflammation levels, and fibrosis progression/remission [83, 84].

The article "Identification of Key Biomarkers and Immune Infiltration in Liver Tissue after Bariatric Surgery" was retracted in 2023. Reasons: unreliable results or conclusions; concerns about the data; concerns about the peer review; concerns about the citations.

With the rapid advance of high-throughput sequencing and bioinformatics analysis, the importance of networks as the presentation of multiple types of biological data, such as protein interactions, gene regulation, cellular pathways, and signal transduction, is increasingly prominent. The importance of nodes in the network could be imputed by examining their network features, which help us identify the central elements of the biological network [85]. CytoHubba, a plug-in from Cytoscape, provides 11 methods of topology analysis based on the shortest path, among which the performance of MCC is better than other methods [86]. WGCNA is a system-biology approach applied to depict gene association according to the interconnectedness of gene sets as well as the correlation between gene sets and phenotypes that contributes to recognizing strongly covarying gene sets and promising treating targets. Module membership, namely, eigengene-based connectivity KME, is used to indicate the association between the gene expression profile and the eigengene of the interested module. Intramodular hub genes at tight junctions have a preference for higher module membership values in modules [87]. Therefore, this study combines the MCC algorithm of CytoHubba and the threshold selection method according to KME values of WGCNA, to determine the hub genes, including SRGN, CD53, EVI2B, MPEG1, NCKAP1L, LCP1, and TYROBP. In order to verify the relevance between hub genes and metabolic liver disease, we obtained and analyzed the mRNA expression level of hub genes using the Attie Lab Diabetes Database and found that in comparison with the lean group, the LCP1 expression level in liver tissues of obese mice at 4 and 10 weeks was significantly upregulated.

The article "Identification of Key Biomarkers and Immune Infiltration in Liver Tissue after Bariatric Surgery" was retracted in 2023. Reasons: unreliable results or conclusions; concerns about the data; concerns about the peer review; concerns about the citations.

Lymphocyte cytosolic protein 1 (LCP1), a member of the family of actin-binding proteins, was previously thought to be specifically expressed in the hematopoietic cell lineage. However, a growing number of studies have shown that LCP1 was detected in many types of human malignant cells of nonhematopoietic origin, suggesting that it could be induced to express in tumorigenesis in solid tissues [88]. More interestingly, LCP1 was reported to be a factor in preventing fat Browning in white fat cells. LCP1 deficiency resulted in increased lipid catabolism, inhibition of fat production, and induction of fat Browning [89]. In a genome-wide association study (GWAS), the mRNA level of LCP1 in liver tissues of NAFLD patients was dramatically elevated (300%) in comparison with the control group (*P* < 0.05). The association between LCP1 single nucleotide polymorphism and NAFLD indicated that LCP1 might be involved in the incidence of NAFLD. Miller et al. adopt proteomic techniques to describe the proteome of NAFLD and found that LCP1 performed well in distinguishing the disease state from the control group, single steatosis from NASH, and fibrosis grading [90], which was consistent with our findings. Therefore, LCP1 has promising application prospects as a noninvasive marker of NAFLD/NASH, which is expected to replace liver biopsy to distinguish NAFLD disease stage and detect liver fibrosis degree.

To further investigate the role of immune cell infiltration in NAFLD, CIBERSORT was applied to comprehensively evaluate the immune infiltration in liver samples before and after bariatric surgery. We found that the postoperative group generally contained a lower proportion of M1 macrophages (*P* = 4.2*E* − 03). The M1 macrophage is a polarized form of Kupfer cells (KCs). Activation of KCs displays a critical impact on the occurrence and progression of NAFLD, owing to the fact that depletion of these cells can reduce insulin resistance, inflammatory development, and even fibrosis [60]. KCs exhibit different forms of polarization depending on the local stimulatory microenvironment [91], including classically activated M1 and another M2 phenotype. The M1 phenotype has traditionally been considered proinflammatory and the M2 as “immunomodulatory,” because the latter is involved in wound healing and anti-inflammation. However, this bisection concept does not fully reflect the complex biological function of macrophage subpopulations, because in some cases, KCs may express markers representing both M1 and M2 differentiation [92].

The article "Identification of Key Biomarkers and Immune Infiltration in Liver Tissue after Bariatric Surgery" was retracted in 2023. Reasons: unreliable results or conclusions; concerns about the data; concerns about the peer review; concerns about the citations.

By analyzing the correlation between LCP1 and immune cells, it was found that LCP1 was significantly positively correlated with memory B cells as well as M1 macrophages and negatively correlated with CD8 T cells as well as regulatory T (Treg) cells. As mentioned above, both innate immunity (neutrophils, macrophages, NK cells, etc.) and adaptive immune system (B cells and various types of T cells) participate in the pathogenesis of NAFLD/NASH, interacting with each other. Neutrophils exacerbate the ongoing inflammatory state by enhancing macrophage recruitment and interaction with antigen-presenting cells [93]. The M1 macrophage is commonly characterized as “proinflammatory” and promotes lymphocyte recruitment and activation by releasing IL-12, IL-23, and lymphocyte chemokines [94]. The cytokine network produced by TH1, TH17, and CD8+ lymphocytes provides a potent stimulus for the activation of M1 macrophages, thus creating further occurrence of liver inflammation [46, 95, 96]. Liver NK cells exhibit different immunophenotypes and functional characteristics from peripheral NK cells, of which the role of participating in NAFLD is not completely clear [97]. However, some studies discovered that liver tissues in NASH rat models showed decreased cytotoxic activity of NK cells [98]. The main effect of regulatory T (Treg) cells is to prevent autoreactions to autoantigens and to avoid overactivation of effector T cells and subsequent tissue damage during immune responses [99]. A fall in the number of liver Treg cells has been reported in animal models of NAFLD [100, 101]. B cells were observed to be activated during an episode of steatohepatitis and mature into plasma blasts and plasma cells in NASH patients and mouse models [49, 102]. Therefore, it is reasonable to speculate that LCP1 overactivated M1 hepatic macrophages and B lymphocytes by inhibiting Treg cells and regulating T effector cell functions, thereby contributing to the occurrence and progression of NAFLD/NASH. Of course, further research is required to elucidate the complex interactions between genes and immune cells.

There are some limitations to our study. First, the data performed in our research was obtained from public databases; thus, the quality cannot be accurately assessed. Second, the scoring system applied to evaluate the histological characteristics of NAFLD may have some subjective factors, which may lead to a certain baseline deviation between the two sets of data. Finally, the sample size enrolled into the analysis is relatively small, which may fail to cover the influence of race, geography, and other factors on the whole analysis and conclusions in this study.

The article "Identification of Key Biomarkers and Immune Infiltration in Liver Tissue after Bariatric Surgery" was retracted in 2023. Reasons: unreliable results or conclusions; concerns about the data; concerns about the peer review; concerns about the citations.

## 5. Conclusions

While limitations remain, we argue that bariatric surgery reduces inflammation or even shifts NAFLD from a “proinflammatory” state to an “anti-inflammatory” state, reducing cellular stress injury and improving metabolism, thus alleviating tissue damage, which is a key mechanism for NAFLD remission after bariatric surgery. We screened out the differential genes before and after surgery and revealed the possible pathways through comprehensive analysis. We then identified LCP1 as perhaps the most critical gene for bariatric surgery to improve liver function and demonstrated its relevance to the innate and adaptive immune system involved in the pathogenesis of NAFLD. More comprehensive researches are required to validate and uncover in-depth mechanisms. These results may identify new potential therapeutic targets to relieve NAFLD that are expected to effectively improve clinical remission of NAFLD in a noninvasive manner.

## Figures and Tables

**Figure 1:** DEG screening and presentation after bariatric surgery. PCA cluster diagram of gene expression matrix: (a) GSE48452 and (d) GSE83452. Volcano plots of DEGs: (b) GSE48452 and (e) GSE83452. Red points represent upregulated genes and green represent downregulated genes. The screening criteria is |*logFC*| > 0.5 and adj *P* < 0.05. Heat map of DEGs identified in (c) GSE48452 and (f) GSE83452. Venn graph of coexpressed DEGs from the two datasets: (g) 10 DEGs were upregulated; (h) 55 DEGs were downregulated in both two datasets.

**Figure 2:** GO enrichment, KEGG pathway analysis, and GSEA of overlapping DEGs. (a) Gene Ontology (GO) enrichment analysis in terms of molecular function (MF), biological processes (BP), and cell composition (CC). The *x*-axis represents the logarithmic transformation of the *P* value, and the *y*-axis represents the GO terms. (b) Chord diagram shows the distribution of DEGs in KEGG enrichment. The left side of the diagram shows the symbol of DEG (whose logarithmic transformation of *P* value is mapped by color scale), and the color line indicates the involvement of DEGs in the KEGG enrichment pathway. GSEA plots show the six most significantly enriched gene sets in the prebariatric surgery group of the GSE48452 (c) and GSE83452 (d) datasets, as well as the three most significantly enriched gene sets in the postbariatric surgery group of the GSE83452 dataset (e). Gene sets are displayed in different colored curves, and the corresponding items are shown below the curves.

**Figure 3:** PPI network and pathway and process enrichment analysis of overlapping DEGs. (a) PPI network construction for overlapping DEGs. Different colors represent different modules where genes were closely connected. (b) Graph shows pathway and process enrichment analysis with best *P* value score to each MCODE component.

The article "Identification of Key Biomarkers and Immune Infiltration in Liver Tissue after Bariatric Surgery" was retracted in 2023. Reasons: unreliable results or conclusions; concerns about the data; concerns about the peer review; concerns about the citations.

**Figure 4:** Construction of WGCNA and screening of interested modules. (a) Heat map displayed the correlation between gene modules and phenotypes. Color depth represents the strength of correlation, and the text explicated correlation coefficient and significant *P* value. (b) Vector graph displayed the relationship between phenotypic characteristics and the module and gene expression within the module. The horizontal axis represented the correlation between the phenotypic features and the red module, and the vertical axis represented the correlation between the phenotypic features and the gene expression in the red module.

**Figure 5:** Identification and validation of hub genes. (a) Venn diagram showed the hub genes determined by MCC algorithm and KME values. (b) The expression of genes including TYROBP, LCP1, CD53, EVI2B, MPEG1, and NCKAP1L. LCP1 expression was significantly upregulated in obese mice compared with the lean group. ^∗∗∗^*P* < 0.001, ^∗∗^*P* < 0.01, and ^∗^*P* < 0.05.

**Figure 6:** Immune infiltration of liver tissue and the correlation between LCP1 and infiltrating immune cells. Violin plot showed the differences regarding immune infiltration of liver tissues before and after surgery in GSE83452 (a). Heat map of correlation of 22 types of immune cells in the preoperative samples of GSE83452 (b). Accumulative bar diagram displayed the relative proportions of immune cells in each sample in the GSE83452 (c) datasets. Green represented a positive correlation, while blue represented a negative correlation. The size of the colored squares represented the strength of the correlation. Correlation between LCP1 and infiltrating immune cells in GSE83452 (d). Dots to the right of *x*-axis zero indicate a positive correlation, while to the left indicate negative. The size of dots represents the strength of the correlation. *P* values were listed on the right side of the vertical axis. ^∗∗∗^*P* < 0.001, ^∗∗^*P* < 0.01, and ^∗^*P* < 0.05.

## Data Availability

All the data used to support the research are included within this article.
